RETRACTED

# Construction of Intelligent Substation-Optimized Networking Communication Network Based on Source-Network-Load Interaction Environment

**DOI:** 10.1155/2022/4730233

**Published:** 2022-09-28

**Authors:** Yubin Lin, Xiaofei Ruan, Jiyu Li, Xiaoyu Huang, Dishan Yang

**Affiliations:** Department of Evaluation Center, Economic and Technological Research Institute of State Grid Fujian Electric Power Co. Ltd, Fuzhou 350000, Fujian, China

## Abstract

Smart grids, which possess flexibility, cleanliness, safety, economy, and friendliness, have drawn a lot of attention from all over the world in an era of rapid social and economic development, power technology change, and energy and environmental constraints. However, there are still issues with the design, installation, and operation of smart substations, such as insufficient LAN integration, difficulty quantifying network performance, and inability to keep track of communication. The basic meaning and key technologies of substation communication standards are used as the research object in this paper, and the basic attributes of substation data flow, such as source, type, and function, are qualitatively analyzed. The mathematical model that is most closely fitted is 2.8% more effective. The research object is the topology of the process bus. Through the comparison of various solutions, including star topology, ring topology, bus topology, and mesh topology, the advantages and disadvantages of each topology networking scheme are revealed along with the particular functional requirements of the substation process layer. Further discussion is given to the crucial topology-related technologies of network congestion and flow control.

## 1. Introduction

Global energy scarcity and environmental pollution have emerged as two of the most pressing issues facing all nations in the world as a result of the accelerating growth of the global economy and the rising demand for energy. The world is now primarily concerned with energy conservation and wise use, and the conventional power system based on fossil fuels is currently facing significant difficulties. The operation and upkeep of the communication network is primarily dependent on “doing its best” performance, and suitable network optimization control strategies and methods for the power system are lacking. Only a large number of redundant pieces of equipment, which wastes resources, can ensure reliability. Countries all over the world have committed significant financial and human resources to conducting research on smart grids in response to this new challenge. To improve the theory of source-grid-load interaction coordinated control and realize grid-friendly and user-satisfactory coordinated and optimal smart grid operation, comprehensive acquisition of power grid data and systematic research on smart grid will undoubtedly be of great significance. It can not only achieve the power grid's safe and effective operation, make effective use of energy, and meet the nation's major strategic needs but it can also significantly affect environmental protection, the development and use of new energy, and the encouragement of the nation's economy's sustainable and harmonious growth.

RETRACTED

Many nations now conduct research on intelligent substations. The distributed implementation of complex functions is made possible by increased computing capacity and recently acquired communication infrastructure in thousands of secondary substations. A few years ago, this was unimaginable. For substation automation equipment, Faschang et al. proposed a flexible and modular software ecosystem that can meet these needs [1]. Liu et al. proposed a substation area protection relay, which can reduce the overall coordination degree, in an effort to address the inherent flaws of the conventional backup protection system [2]. In smart substations, Zheng et al. was the first to propose a high-reliability optical process level network scheme with all-optical passive edge nodes [3]. The communication network in substations has recently received increased attention from all parties due to the emergence of smart substations. Based on the communication network of smart substations, Liu thoroughly examined the process and execution process of various business chains [4]. The aforementioned researchers and analysts have done research and analysis on smart substations, but they have not combined the source-network-load interaction model to explain, and their work is somewhat irrelevant.

A new model for understanding power systems is source-grid-load interaction background. However, there are some restrictions. Augmented reality in the classroom has grown to be an intriguing research topic in education. A multimodal interaction algorithm based on augmented reality that uses visual and haptic feedback was proposed by Xiao to address these problems [5]. Distributed energy supply and natural gas industrial IoT based on trusted transactions have emerged as one of the hottest research hotspots in the energy sector as a result of the development of energy interconnection and the constant rise in natural gas consumption. To address the drawbacks of the centralized energy supply architecture, Miao et al. proposed an Internet of Things (IoT) architecture for the natural gas industry based on blockchain and artificial intelligence [6]. A method for anticipating the load noise of high voltage transformers was put forth by Kim et al. The electromagnetic force is produced when the transformer is loaded by the interaction of the electric and magnetic fields. This force, known as the Lorentz force, can result in load noise in the transformer by causing vibrations in the winding structure [7]. These open systems are incredibly complex, but their programming abstractions help the client layer. Different capabilities can be provided by third-party applications at the client layer, opening up business opportunities for optimization-as-a-service. For offline planning, online configuration, and orchestration of SDN/NFV networks, Garrich introduced an open source optimization software initiative [8]. The aforementioned researchers performed experimental analysis on the source-network-load interaction model without disclosing the experimental methodology and should be supplemented on this basis going forward.

RETRACTED

The originality of this paper is that it uses the data flow of a smart substation as its research subject and builds a simulation platform for the network communication system of the smart substation based on OPNET. The technical viability and superiority of implementing a dual-star topology along with a VLAN strategy in an intelligent substation network communication system—which is superior to other technologies—is shown from the perspective of network throughput and delay indicators.

## 2. Method Based on the Piecewise Function Model under the Source Network Load

The purpose of synergy between renewable energy and conventional energy, transmission grid and distribution network, and the controllable load is to achieve safe, economical, and environmentally friendly grid optimization scheduling [9]. Its analysis and optimization methods involve multiple disciplines, which are interrelated and support each other.

### 2.1. Uncertainty of Wind Power Based on the Piecewise Function Model

Wind energy has attracted much attention because of its huge potential, mature technology, and green environmental protection, and its installed capacity is much higher than that of other renewable energy sources such as solar energy [10]. The basic structure of the wind turbine is shown in Figure 1.

Because the natural wind speed changes greatly, the operation mode of the wind power generation system generally changes according to the change of the wind speed, and the output model of the generated power can be described by the piecewise function according to the change of the wind speed. The relationship between wind power, output power, and wind speed is as follows:

(1) $$\begin{array}{c} h_{m}=\left\{\begin{array}{c} 0\\ \frac{n-n_{w}}{n_{i}-n_{w}}\\ h_{t} \end{array}.\right) \end{array}$$

It can be seen from formula (1) that the output of wind power depends on the wind speed, which is unstable in time, unbalanced in space, and has certain seasonal distribution characteristics.

RETRACTED

When the wind speed is a discrete random variable, the wind speed can be divided into several wind speed segments within [*o*, *g*], which are [0, 1], [1, 2],…, [*g* − 1, *g*]. Among them, *G*is the maximum local wind speed. Counting the duration *p*_*t*,*r*_ (*t*=1,2,…, 11; *r*=1,2,…, *m*) corresponding to each wind speed segment in each month, the probability  *h*_*r*_ (*r*=1,2,…, *m*) of each wind speed segment occurring within one year can be obtained, which can be expressed as

(2) $$\begin{array}{c} h_{m}=\frac{1}{8670}\sum_{t=1}^{11}p_{t,r}. \end{array}$$

The empirical distribution function of regional wind speed corresponding to formula (2) is given as

(3) $$\begin{array}{c} H\left(d\right)=\sum_{i=1}^{n}f_{i}. \end{array}$$

When the wind speed is a continuous random variable, its probability density function can be expressed as

(4) $$\begin{array}{c} h\left(d\right)=\frac{w}{q}{\left(\frac{d}{w}\right)}^{q-1}\text{exp}\left(-{\left(\frac{d}{w}\right)}^{q}\right). \end{array}$$

The analytical expression of the cumulative distribution function is

(5) $$\begin{array}{c} H\left(d\right)=\int_{-\infty }^{d}h\left(d\right)dd,\\ =1-\text{exp}\left(-{\left(\frac{d}{w}\right)}^{q}\right). \end{array}$$

Among them, *w* > 0 is the scale parameter, and *q* > 0 is the shape parameter, which is related to the specific wind farm location.

The uncertainty of the above-mentioned changes in wind energy resources makes the output power of wind farms to have strong randomness. When the grid is connected to determine the dispatching operation plan of the system, it is generally necessary to determine the fluctuation range of the output of a certain wind farm output trend and to determine the boundary value of the wind farm output with a certain degree of confidence [11]. In general, it can be expressed as

(6) $$\begin{array}{c} H_{m-}=\text{max }\left\{\beta \left|\right)H_{t}\left(H_{w}\geq \beta \right)\geq \alpha \right\},\\ H_{m+}=\text{min }\left\{\gamma \left|\right)H_{t}\left(H_{w}\leq \gamma \right)\geq \alpha \right\}. \end{array}$$

### 2.2. Unit Start-up Cost Based on the Piecewise Function Model

Since the start-up consumption of the unit is nonlinear, it needs to be linearized in the process of unit combination optimization. The usual processing method is to use a piecewise function to represent it, as follows.

The start-up cost of the unit can be expressed as

(7) $$\begin{array}{c} D_{f,i}=\left\{\begin{array}{c} D_{f,i}^{\text{hot}}\\ D_{f,i}^{\text{cold}} \end{array}\right). \end{array}$$

RETRACTED

### 2.3. Interaction Mechanism Based on Physical Characteristics of the Load and Electricity Consumption

After the large-scale access of electric vehicles, they will serve as the main high-power electricity load of users. Effective analysis of battery physical characteristics and performance and energy estimation that can participate in the interaction are the basis for its participation in the interaction between the source, the network, and the load [12].

#### 2.3.1. Physical Characteristics and Model of Electric Vehicle Battery Charging

Lithium batteries are also the main power batteries for modern electric cars. The common battery model consists of a controlled current source and a constant value internal resistance in series, and for lithium batteries, the model also includes

(8) $$\begin{array}{c} M=W_{0}-\frac{KTI}{0.2T+P\left(r\right)}-\frac{KTP\left(r\right)}{T-P\left(r\right)}+Bd-TY,\\ p\left(r\right)=\left(1-\frac{Q_{0}}{100}\right)T+\int_{0}^{1}Ydr. \end{array}$$

#### 2.3.2. Electric Vehicle Daily Driving Power Consumption Model

The driving behavior of electric vehicles is the main reason for their power consumption, and the power consumption is closely related to the driving distance. The speed of the vehicle at each moment can be regarded as a random variable, and the speed at different times obeys a normal distribution, then the electric vehicle power consumption can be expressed as

(9) $$\begin{array}{c} W_{t,r+1,m}=W_{t,r,m}-\frac{W_{total}}{G_{total}}G_{t,r,m}. \end{array}$$

Among them, *G*_*t*,*r*,*m*_ is the distance traveled in the *t*period, and the running distance of the electric vehicle in each period can be determined according to the travel time, the distance distribution of a single trip, and the speed distribution. *G*_total _is the cruising range when the vehicle is fully charged, and *W*_total _is the power when the battery is fully charged.

#### 2.3.3. An Interactive Electric Vehicle Battery Remaining Power Analysis Model

The energy of electric vehicles participating in grid interaction comes from the power battery, and the analysis of the remaining battery power is the basis for whether it can participate in the interaction. The calculation formula of the ampere-hour metering method is

(10) $$\begin{array}{c} DTY=DTY_{0}-\frac{1}{F_{N}}\int_{r_{0}}^{r}\beta E\text{d}r. \end{array}$$

Among them, *DTY*_0_ is the initial remaining capacity of the battery at the time of *r*_0_, and the principle of the open circuit voltage method is as follows:

(11) $$\begin{array}{c} DTY=\frac{M_{0}-c}{d-c}, \end{array}$$

where *M*_0_ represents the open circuit voltage of the battery, *d*represents the open circuit voltage of the battery when the battery is fully charged, and*c*represents the open circuit voltage of the battery when the battery is fully discharged.

RETRACTED

### 2.4. Optimization-Based Interactive Optimization Method

The system solutions implemented by grid interaction mainly include source-source complementarity, source-grid interaction, grid-load interaction, and source-load interaction, as shown in Figure 2.

The optimization problem can generally be expressed in the following mathematical form:

(12) $$\begin{array}{c} \min k\left(a\right),a\in A\subset M^{n}. \end{array}$$

The constraints are as follows:

(1) Constraints on the number of fans, the number of photovoltaics, and the number of batteries:
  (13) $$\begin{array}{c} \left\{\begin{array}{c} 0\leq M_{n}\leq M_{n,\text{max}},\\ 0\leq M_{e}\leq M_{e,\text{max}},\\ 0\leq M_{t}\leq M_{t,\text{max}}. \end{array}\right) \end{array}$$
Among them, *M*_*n*,max_,  *M*_*e*,max_, *M*_*t*,max_ stands for wind turbine, photovoltaic, and energy storage battery, respectively [13].
(2) Constraints on the change of the power of the energy storage battery:
  (14) $$\begin{array}{c} \left\{\begin{array}{c} M_{t,\text{min}}<M_{t,dty}<M_{t,\text{max}},\\ M_{t}<M_{t,\text{max}}. \end{array}\right) \end{array}$$
(3) The distribution network power flow equation constraints of distributed energy:
  (15) $$\begin{array}{c} M_{t}\left(r\right)=H_{m}\left(M_{jq}\left(r\right),P_{EYS}\left(r\right),B\left(r\right)\right). \end{array}$$
(4) Distributed power output constraints:
  (16) $$\begin{array}{c} M_{jq}^{\text{min}}\leq M_{jq}\left(r\right)\leq M_{jq}^{\text{max}}. \end{array}$$

## 3. Communication Network Simulation of Intelligent Substation Networking

### 3.1. Network Congestion

1. Source, network, and load interaction information:The continuous development of information access and transmission technology makes it possible to interact with energy resources on the power generation side and the load side, and it also provides new ideas for eliminating the uncertainty of renewable energy output. Through the two-way information flow, the load side can better participate in the power balance, and the power generation side can respond quickly to real-time information, making the realization of the dispatch plan more flexible. Compared with the relatively complete power infrastructure, the information access and transmission technology suitable for the interaction between the source, network, and load are still being perfected. Existing research results support a large amount of information exchange in random access environment, especially the reliable transmission of time-sensitive information and diverse services. Therefore, the energy estimation and benefit analysis that the load side can participate in interaction has become one of the hotspots of interaction research.
2. The phenomenon of network congestion:The basic route of data flow communication can be represented, as shown in Figure 3. The source node encapsulates the data information to be transmitted according to certain rules, forwards it through each channel node of the communication network, and transmits it to the destination node. The destination node parses the received message and reads the original content. When the channel capacity matches the number of source nodes and destination nodes, the overall network communication can maintain a good and smart state, with fast data transmission and low or even zero packet loss rate in the intermediate links [14]. An extreme case of network congestion is deadlock. The description of the congestion phenomenon is shown in Figure 4.
3. Reasons for network congestion:Network communication itself is a dynamic problem, and the imbalance of resource allocation is another major factor causing congestion, as shown in Figure 5.

RETRACTED

### 3.2. Simulation of Smart Substation Network Performance

#### 3.2.1. Simulation Model

In this paper, the network simulation model of the open-type distribution substation based on IEC 61850 is established in the simulation system. Compared with the previous research, a complete data flow object is established. The network adopts a star structure, and information is shared through switches. As shown in Figure 6, the whole system includes 20 bay models and a synchronous clock device [15]. The switch communication network is 100 Mbps. Each bay includes 1 process bus switch, 3 centralized units, 3 intelligent isolation switches, 3 grounding switches, and differential protection units, interbay control units, and line protection units.

According to the idea of IEC 61850 information layering, the specific communication behavior of the simulation model is as follows:

1. The centralized unit mainly conducts sampling and continuously broadcasts the sampled value message within this interval. The sampling rate is 6 kHz. The transmission frequency of the message is equal to the sampling rate, and it is transmitted in the Ethernet format.
2. The flow starts 50 s after the simulation starts.
3. The protection unit starts to continuously send a broadcast message with a frequency of 2 kHz for 10 ms after 72 s from the start of the simulation.
4. The bay layer control unit starts to simulate the actuator sent to the ISG in the nacelle after 80 s and sends it to the other two control protection units with the same time interval message to simulate functional interlocking.
5. The engineer station generates these data through the business to observe the network performance and randomly sends a message to the main control unit of the substation 120 s after the simulation starts, using the TCP protocol, and the duration is 1 s. The random information such as protection action and fault recording is uploaded to the substation in the simulated bay layer [16]. The simulation time is 150 s, and the switch adopts the way of full storage and forwarding. The synchronous clock message period sent by the station-level synchronous clock device is 1 s, and the length is fixed to 72 bytes. A shielded twisted pair cable is present with a data link length of 100 m in the network. During the emulation process, the priority of all packets is set to be the same.

RETRACTED

#### 3.2.2. Substation Network Communication and Result Analysis

We can obtain the performance index of the network by analyzing the network nodes. The BCU is the heaviest network load in the process layer, and almost the main data flows here. Therefore, the network performance can be obtained by analyzing the throughput and packet arrival delay of the BCU network traffic.

First, verifying the impact of VLAN technology on network performance is done. In the simulation model described above, two intervals are selected as target intervals. When VLAN technology is not used for division, all devices are in one subnet, and the network throughput of BCU is shown in Figure 7(a). The two intervals are divided into VLANs, and each interval is divided into a VLAN. The simulation results are shown in Figure 7(b). The BCU network load simulated by the two is quite different, and the load of using VLAN technology is only about one when it is not used. Therefore, it is concluded that the use of VLAN technology can reduce the load rate of the network, reduce the risk of network congestion, and effectively improve the real-time performance of the network.

The simulation result of process layer communication is shown in Figure 8. Although there is a certain amount of jitter in the transmission of various types of messages during the simulation process, they are all within the allowable range and are relatively stable throughout the simulation process [17]. The load of the BCU accounts for the vast majority of the entire network load. As can be seen from Figure 8, it is 3 Mbps, which only accounts for 3% of the 100 Mbps Ethernet, and it is estimated that the traffic of other network nodes will not be very high. By counting data packets of all nodes, there is no packet loss.

RETRACTED

The simulation results of substation layer communication are shown in Figure 9. Under normal conditions, the network load is only 5% of the 100 Mbps Ethernet bandwidth, and even if there are unexpected events such as failures, it will not exceed 40% [18]. Through the statistical data tracking file, the data packets during the entire simulation process were calculated, and no packet loss occurred. Through the above simulation, it can be seen that the performance of the substation communication network established in this paper meets the IEC 61850 standard. The real-time performance of the network can be improved by dividing VLANs.

### 3.3. 110 kV Intelligent Substation Network Structure and the Networking Scheme

#### 3.3.1. Analysis of the Network Structure of the Intelligent Substation System

The DL/T860 standard defines the substation automation system model. According to the functions of the substation IED equipment, the data exchange methods between the functions of each layer are mainly as follows:

1. Exchange protection and control data through the GOOSE service so that equipment from different manufacturers can exchange data under a unified standard.
2. Between the spacer layers, the fast and direct exchange of data is generally realized through the GOOSE service.
3. The process layer mainly includes the following two interfaces: sensor (TA/TV) interface and actuator (smart switch and transformer).
4. The establishment of the DL/T860 model from the station control layer to the distant place has not been perfected, and most of them still use traditional methods to exchange data. The typical wiring diagram of the station control building and the process layer is shown in Figure 10:

The station control layer uses 24 electrical + 2 optical switches, a central switch, 10 kV interval, single star network structure, and 110 kV switch interval [19]. The station control layer is generally configured with four switches, and the specific number can be appropriately increased or decreased according to the scale of the substation, as shown in Figure 11.

110 kV process layer GOOSE, SV combined network, 35 (10) kV process layer is not networked. The process layer switch adopts 16 optical port switches. In the process layer, one central switch is set for each main transformer, and there is one switch for every four intervals of 110 kV. The process layer is generally configured with five switches, and the specific number can be appropriately increased or decreased according to the scale of the substation. According to the different information transmission paths and the degree of network integration optimization, the commonly used networking forms of existing smart substations are shown in Table 1:

The networking form 2 allows for the direct transmission of the SV and GOOSE data needed by the automation application to the station control layer network via optical fiber, and the relevant manufacturers also supply the technology to the station control layer network via the bay layer IED. This is something that needs to be highlighted.

RETRACTED

#### 3.3.2. Analysis of Key Technologies Using Three Layers and One Network

*(1) Network Traffic Analysis*. In the three-layer one-network solution, the bay layer and the process layer IED are further optimized and integrated, and the bay function is complete and autonomous. Interinterval interlocking GOOSE and other interinterval back-moving or jumping alarms (such as failure start, backup automatic switching, and main transformer backup protection jumping segment) are transmitted through the station control layer network. The SV information of each bay is “transmitted” through the bay layer IED to the network packet analysis and advanced applications of the integrated platform.

The information transmitted by the station control layer network after the three-layer one network includes (SV, GOOSE, IEEE1588, and MMS) messages. The length of the MMS message is generally within 500 bytes, and the transmission interval is 100 ms. Even if the maximum packet length of Ethernet is 1518 bytes, the MMS packet rate of the device port at the bay layer is about 0.12 Mbps. The traffic is very small, and according to the IEC 61580 specification, the priority of MMS is low, and the traffic can be limited by setting, so the occupation of network bandwidth by MMS packets is also very limited [20]. Based on the above two points, GOOSE packets and SV packets can be mainly considered in traffic analysis.

There are some uncertain lengths in the IEC 61850-9-2 sample value packet, which is related to the number of ASDUs. The maximum length of each SV message is 171 bytes, and it is sent to every 250US. On comprehensive consideration, the protection device with the largest single-port flow in this paper is the 110 kV busbar protection device, and 110 kV is increased by eight intervals in the final period.

*(2) Real-Time Analysis of Network Packets*. The characteristics and requirements of intelligent substation network transmission messages are shown in Table 2:

From the analysis of the above table, it can be known that the SV (sampled value) packets have relatively large traffic, but the packet traffic is very stable. The small average traffic is the GOOSE message, but the burst traffic is also relatively large. The MMS message is with the smallest average traffic, but the burst traffic is very large, and the above message is a total network transmission. If no effective preventive measures are taken, the reliability and real-time performance of SV and GOOSE messages will be affected by burst MMS messages. These messages have great relevance to protection [21]. Therefore, when the communication network is “three networks and one layer,” the GOOSE message related to the automation function should be set to a lower priority. In order to reduce the impact on protection, the GOOSE message and SV message must be set to a higher priority to reduce the impact on system reliability and real-time performance.

RETRACTED

The process layer intelligent component is an integrated design device, which is directly connected to the point-to-point optical fiber of the bay layer equipment. SV and GOOSE are used for common cable transmission, which can save 50% of optical cable connections, thus effectively simplifying the workload and investment of secondary wiring. The reason why SV and GOOSE can jointly transmit is because the transmission characteristics of the two kinds of messages are different. The traffic of SV packets is stable and sent regularly. The stable flow of GOOSE messages is small, the burst flow is large, and the real-time requirement of sudden change transmission is high. The minimum transmission interval is 1 ms, and the transmission interval is gradually lengthened. The message is maintained normally, and the transmission interval can reach 5 s.

#### 3.3.3. Network Configuration and Implementation

*(1) Overall Scheme of Network Configuration*. According to network traffic analysis and comprehensive consideration, the 110 kV substation project has the following characteristics:

① The equipment on the partition layer is placed in the intelligent control cabinet. Among them, the 110 kV line, subsection, and main transformer backup protection have completed the integration of the process layer and the interval layer;
② 35 kV/10 kV adopts the integrated device of protection, measurement and control, wave recording and measurement, and the switchgear is installed on-site, and the integrated device is directly connected to the station control layer network. Under the premise of ensuring reliability and real-time principle, it combines the characteristics of substation engineering in 110 kV area. For the sake of economy, the 110 kV substation project was decided to be designed as “three layers and one network,”in which the interval layer and the process layer are directly connected with optical fibers, and no process layer switches are set up, and the optimization of network technology is added. This satisfies the real-time requirements of a large number of data streams on the network.

*(2) Network Implementation Plan*. Only one integrated information platform machine is configured at the station control layer. As a unified and unique information platform in the station, it integrates the functions of the host and operator station, the five-proof workstation, and the total station standby operation and provides advanced application functions such as sequence control and intelligent alarm. The interval layer is composed of independent subsystems to protect the direct sampling and direct jumping. The network structure adopts a single star network structure, and the network switches are configured according to their functions.

RETRACTED

One 1000 M switch is installed as the central switch and two 100 M switches are installed in the main control room group screen. Among them, the 1000 M central switch is equipped with 8 electrical ports and 8 optical ports. The electrical port is mainly used to connect the station control layer equipment, and the optical port is mainly used for switch cascade; the two 100 M switches are each equipped with 12 optical ports and 4 electrical ports. The optical port is used to connect 110 kV spacer layer protection measurement and the control device. The 110 kV busbar protection device, integrated power supply, public monitoring and control, and other common and ingenious equipment are connected to the electrical port of the switch through CAT-5E shielded twisted pair cables.

*(3) Technical Requirements for Network Switches*. The intelligent substation replaces the traditional secondary circuit with information network transmission, so it puts forward very high requirements for the networking switch. In particular, strict requirements are put forward for the real-time nature of data transmission, and switches are required to have functions such as preferential transmission for part of the replayed data. An industrial-grade switch certified by KEMA should be used, and it should have at least the following functions.

① Priority transmission function: According to the pressure EE802.1 P standard, the serial number QS of the priority Ethernet packet header can be added to identify the quality of service, and the priority of switching forwarding is based on the principle of weight or traffic distribution.
② Under the mainstream standard of IEEE802.1Q, there are several VLAN technologies based on switch ports, MAC addresses, and protocols.
③ Dual power supply function: In order to ensure reliability, each switch should have two channels of DC power supply, and it has the corresponding fault alarm signal output function.
④ With IEEE1588 time setting function: PTP precision time protocol is used by the combination of hardware and software, which can achieve the time synchronization accuracy of microsand level. Industrial Ethernet switches need to specifically support end-to-end.

RETRACTED

### 3.4. Experimental Results

In this chapter, according to the data flow sending and receiving characteristics of the actual physical equipment of the smart substation, the OPNET simulation software is used to establish the dynamic data flow simulation platform of the smart substation. According to the corresponding relationship between the actual physical equipment and the data flow mathematical model, the qualitative selection of the distribution function and the quantitative parameter configuration are carried out on the substation simulation platform. For different scenarios, such as 10 M and 100 M communication links, four expansion modes such as single-star, double-star, ring, and mesh topology are seen; GOOSE packets and SV packets are divided into networks and shared networks, before and after using VLAN technology, etc., and a series of comparative experiments were carried out. Results of each group of experiments are summarized as follows:

1. The basic characteristics of the data flow of the smart substation are qualitatively analyzed, and the data volume of the GOOSE and SV messages of the smart substation is quantitatively estimated.
2. The network topology of the process layer is analyzed, and the advantages and disadvantages of each scheme are analyzed. The phenomenon and causes of network congestion are discussed emphatically, and the corresponding control strategies are proposed.
3. The network simulation software OPNET is used to build the simulation platform model of the network communication system of the intelligent substation.
4. This work studied the influence of single-satellite mode, double-satellite mode, and ring network topology mode on network performance differences.

## 4. Conclusion

Communication infrastructure and technology have gradually improved, thanks to smart grid. A new wave of new energy development has taken on this theme as a result of the transformation of the conventional power grid. The construction of pilot projects and the development of new equipment are currently the two main issues hindering the development of smart substations. There are not many studies on the networked platform that are suitable for smart substation nodes or even the entire power system backbone network's communication architecture system and performance analysis. This makes it difficult to advance and scale business applications. Although Ethernet technology has been introduced to the power sector, there has not been a significant amount of integration. The data flow of an intelligent substation is therefore used in this paper as the research object, and the network performance is thoroughly examined using a variety of mathematical analysis techniques and software simulation techniques. It is also adopted to combine theoretical analysis with simulation experimentation and to conduct data flow analysis. The efficiency of the intelligent substation network communication system using the dual-star Qiaopu in conjunction with the VLAN technology scheme increased by 2.8 percent, proving its viability and superiority. It improves the research strategies and equipment used in the intelligent substation network communication, which has some scholarly value and engineering-related practical significance.

RETRACTED

## Figures and Tables

**Figure 1:** Basic structure of a wind turbine.

**Figure 2:** Grid interaction implementation diagram.

**Figure 3:** The transfer process of the data flow.

**Figure 4:** Throughput and response time as a function of load. (a) Throughput as a function of load. (b) Latency as a function of load.

**Figure 5:** Unbalanced resource distribution.

**Figure 6:** Smart substation communication simulation model.

**Figure 7:** Using the VLAN emulation effect. (a) Without VLAN. (b) With VLAN.

**Figure 8:** Message transmission characteristic diagram.

**Figure 9:** Substation communication simulation results.

**Figure 10:** Typical wiring diagram of the station control layer.

**Figure 11:** Typical wiring diagram of the process layer.

**Table 1:** Networking forms of smart substations.

	For protection		Automation application		MMS
	SV	GOOSE	SV	GOOSE	
Form 1	Point-to-point fiber		Process level network		Station control layer network
Form 2	Point-to-point fiber		Station control layer network		
Form 3	Process level network				Station control layer network

**Table 2:** Real-time requirements for network packets.

	Average traffic per device (Mbps)	Burst traffic per device (Mbps)	Real-time requirements for messages (Mbps)
SV message	5.5	5.5	<3.5
Protection-related GOOSE messages	<0.002	3.5	<3.5
GOOSE messages related to automation functions	<0.002	4.5	<498
MMS message	<0.02	98	<498

## Data Availability

The data used to support the findings of this study are available from the corresponding author upon request.
